This article has been retracted.

# Chemokine receptor 7 overexpression promotes mesenchymal stem cell migration and proliferation via secreting Chemokine ligand 12

**DOI:** 10.1038/s41598-017-18509-1

**Published:** 2018-01-09

**Authors:** Ling Liu, Jian-Xiao Chen, Xi-Wen Zhang, Qin Sun, Lan Yang, Airan Liu, Shuling Hu, Fengmei Guo, Songqiao Liu, Yingzi Huang, Yi Yang, Hai-Bo Qiu

**Affiliations:** Department of Critical Care Medicine, Nanjing Zhongda Hospital, School of Medicine, Southeast University, Nanjing, 210009 China

## Abstract

Great interest has been shown in mesenchymal stem cell (MSC) therapy in a wide variety of clinical domains. However, the therapeutic efficiency depends on the proliferation and migration of MSCs. Chemokine receptors are involved in regulating the proliferation and migration to the specific organs of MSCs in different microenvironments. CXC receptor seven (CXCR7), a newly discovered Chemokine ligand 12 (CXCL12) receptor, has organ specificity for tumour migration. We hypothesized that CXCR7 expression affects proliferation and migration of MSCs. In present study, we constructed long-term and stable mMSCs lines overexpressing and suppressing CXCR7 modifications with lentiviral vectors. The transduction efficiencies, mRNA and protein expression of CXCR7 were significantly regulated. CXCR7 gene overexpression promoted mMSCs proliferation and migration, whereas suppressing CXCR7 had the opposite effect. Additional CXCL12 improved the vertical migration of mMSCs. The overexpression of CXCR7 increased the MSC-secreted CXCL12, VCAM-1, CD44 and MMP2 levels, which contributed to the improvement of mMSC proliferation and migration. Therefore, overexpressing CXCR7 improved the proliferation and migration of mMSCs, which may be attributable to the CXCL12 secreted by MSCs, leading to a positive feedback loop for CXCL12/CXCR7 axis. Our results may provide a potential method for improving the treatment effectiveness of mMSCs by overexpressing CXCR7.

## Introduction

Mesenchymal stem cells (MSCs), with their multipotent capacity self-renewal potential, ability to migrate to sites of injury after systemic delivery and lack of immunogenicity^1–3^, have potential for use in treating many diseases, such as acute respiratory distress syndrome (ARDS)^4^. There is a growing body of evidence suggesting that chemokine and chemokine receptors are involved in regulating MSC proliferation in different microenvironments and MSC migration to specific organs.

Chemokine (C-X-C motif) ligand 12 (CXCL12), also termed chemokine stromal cell-derived factor (SDF-1), improves the motility of stem cells predominantly through CXC receptor 4 (CXCR4) and/or CXCR7^5^. In most human acute diseases, such as myocardial infarction and cerebral stroke, CXCR4 has been extensively reported to be overexpressed and has earned considerable attention over the last decade. However, CXCR7 may also participate these disease and the mechanisms by which CXCR7 may participate in CXCL12-associated diseases have not been elucidated^6–8^.

In a previous study, the activation of CXCR7 was found to improve the migration of colorectal cancer cells within the lung but not within the liver^9^, which may indicate that activating the CXCL12/CXCR7 axis in tumour cells could improve the secretion of CXCL12 and promote metastasis to lungs specifically^10^. CXCR7 has a lower expression on the surface of cells; however, has a ten-fold higher affinity to CXCL12 than CXCR4^11^. Moreover, infection and injury may promote the secretion of CXCL12 in specific organs, such as the lung. Therefore, we hypothesize that the overexpression of CXCR7 may have positive effects on mouse MSC (mMSC) proliferation and migration to specific organs.

Considering the low expression of CXCR7^10,12^, it is inefficient to temporarily alter CXCR7 expression with its blockers CCX754 or CCX771, or to induce short-term genetic modification for *in vivo* therapy. Thus, it is necessary to construct MSCs such that the overexpression or suppression of CXCR7 is permanent and stable, as a goal of *in vivo* treatment. What’s more, we used a very similar approach to address a question in regards to the effects of modulation of the beta-catenin/Wnt pathway in stem cells^13^. The aim of this study was to construct mMSCs with long-term and stable CXCR7 regulation via lentiviral vector transduction and to evaluate the effects of CXCR7 overexpression on the proliferation and migration of mMSCs as well as the underlying mechanism.

## Materials and Methods

### Cell culture

Mouse MSCs isolated from the bone marrow of C57BL/6 mice and 293FT cells were obtained from Cyagen Biosciences, Inc. (Guangzhou, China). The identification of mMSCs according to their cell surface phenotypes and their multipotency for differentiation along the adipogenic, osteogenic, and chondrogenic lineages was performed by the supplier, as described by Liu and Cai^13,14^. Either mMSCs or 293FT cells were cultured in a 1:1 mix of Dulbecco’s modified Eagle media/nutrient mixture F-12 (DMEM/F12) (Wisent, Inc., St-Bruno, Quebec, Canada) containing 10% FBS (Wisent, Inc.) and 1% antibiotics (streptomycin and penicillin) and incubated at 37 °C in a humidified atmosphere of 5% CO_2_.

### Lentiviral vector-mediated CXCR7 overexpression and knockdown in mMSCs

mMSCs with passage number 4–6 were used for transduction. The recombinant lentivirus vector over-expressing the murine CXCR7 was constructed by using a CMVIE promoter-dependent lentiviral expression vector^15^. The methods used in the present study were the same as methods we have previously used^13^. Briefly, the full-length coding sequence (CDS) of CXCR7 (NM_001271607, 1088 bp), which was purchased from Hanbio Biotechnology Co., LTD (Shanghai, China), was cloned into the lentiviral expression vector between the CMVIE promoter and ZsGreen, followed by T2A-Puromycin. Finally, the lentivectors pHBLV-CMVIE-CXCR7-ZsGreen- T2A- Puromycin (over-expressing CXCR7) were obtained, and the empty vector pHBLV-CMVIE-ZsGreen- T2A-Puromycin was used as an empty control, termed NC (normal control).

A murine CXCR7 knockdown construct expressing short hairpin RNA (shRNA) targeting endogenous CXCR7 was generated in a lentivirus-based shRNA vector driven by the U6 promoter containing ZsGreen^16^. Target sequences were selected by software available on the Invitrogen website. Additionally, a negative control was generated containing non-specific shRNA (pHBLV-U6-ShRNA- ZsGreen-Puromycin).

The recombinant plasmids pHBLV-CMVIE-CXCR7-ZsGreen-T2A-Puromycin, pHBLV-CMVIE-ZsGreen-T2A-Puromycin, pHBLV-U6-ShRNA-ZsGreen-Puromycin or pHBLV-U6-ZsGreen-Puromycin were separately co-transfected with two packaging plasmids pSPAX2 and pMD2G into 293FT cells at the indicated concentrations using Lipofectamine 2000 (Hanbio Biotechnology) according to the manufacturer’s instruction.

mMSCs (2 × 10^5^/well) were seeded in 6-well cell culture plates, grown overnight and transduced with lentiviral vectors in a minimal volume of medium. Two days after the lentivirus vectors over-expressed the target gene, the stable cell lines were selected with 2 μg/ml puromycin. When all of the non-transfected cells disappeared and isolated colonies began to appear, the colonies with the greatest number of cells were chosen for expansion. A limiting dilution assay was used to obtain transduced cell clones expressing ZsGreen. The mMSCs were cultured in normal culture media for 20 passages after transduction to assay their long-term transfection efficiency. The transfection efficiency of the lentivirus vectors in passage 20 transduced-mMSCs was identified using fluorescence microscopy, and the percentage of ZsGreen-positive cells was determined by flow cytometry analysis using a Becton Dickinson FACS Calibur flow cytometer (FACS Calibur, Becton-Dickinson, Franklin Lakes, NJ, USA).

### RNA isolation and quantitative real-time PCR (qRT-PCR)

Total RNA was extracted from the cells using TRIzol reagent (Ambion, Austin, TX, USA). The 260/280 absorbance ratio was measured to verify the purity and the concentration of the RNA. The qRT-PCR reaction was performed using the SYBR Green Realtime PCR Master Mix (Toyobo Co., Ltd., Osaka, Japan) and the Applied Biosystems (ABI) 7500 real-time PCR system (Applied Biosystems, Inc., Foster City, CA). Relative changes in the gene expression were normalized to the expression of MGAPDH levels and calculated using the 2(^−ΔΔ^Ct) method. The primer sequences used for PCR amplification in our study were designed as Table 1.

**Table 1:** The primer sequence of genes.

Gene	Primer sequence
CXCR7-Q1	5′-TACGACACGCACTGCTACATC-3′ (forward)5′-CTGCACGAGACTGACCACC-3′ (reverse)
CXCR7-Q2	5′-GCCTGGCAACTACTCTGACAT-3′ (forward)5′-AAGCACGTTCTTGTTAGGCAT-3′ (reverse)
CXCR7-Q3	5′-AGCCTGGCAACTACTCTGACA-3′ (forward)5′-GAAGCACGTTCTTGTTAGGCA-3′ (reverse)
CXCL12	5′-AGAGCCACATCGCCAGAG-3′ (forward)5′-TTCAGCCGTGCAACAATC-3′ (reverse)
MGAPDH	5′-GTGGCAAAGTGGAGATTGTTG-3′ (forward)5′-CTCCTGGAAGATGGTGATGG-3′ (reverse)
Actin	5′-ATGTGGATCAGCAAGCAGGA-3′ (forward)5′-AAGGGTGTAAAACGCAGCTCA-3′ (reverse)

### Flow cytometric analysis of CXCR7 expression on mMSCs

The CXCR7 expression on the surface of mMSCs was assessed by flow cytometry analysis. After harvested and washed in PBS, mMSCs were suspended in PBS at a concentration of 1 × 10^6^ cells/ml and then incubated for 60 min with 10 µl of the primary antibody of CXCR7 (PE-CXCR7, biolegend) per 100 µl following analysis with a flow cytometer (BD Biosciences). Then the CXCR7 protein (relative expression) as CXCR7 (PE-A)-positive cells/total cells was calculated.

### Cell proliferation assessment

The proliferation of mMSCs was analysed using Cell Counting Kit-8 (CCK8) (Dojindo Laboratory, Japan) according to the manufacturer’s instructions. mMSCs were seeded in 96-well plates at 5 × 10^3^ cells per well in 100 μl of growth medium. The cells were incubated for 2 h at 37 °C. Absorbance was assessed at 450 nm using a microplate reader (Bio-Tek, USA). The mean optical density (OD) of the three wells in each group was used to reflect the percentage of cell proliferation.

### *In vitro* scratch assay

mMSCs were seeded in 6-well culture plates. When the cells reached approximately 100% confluence, a scratch was made with a 10 μl sterile pipette tip, and the cells were cultured in serum-free DMEM/F12 for an additional 24 h^17^. The images of the wound were recorded using a light microscope immediately after scratching and 18 h later. The horizontal migration abilities of the cells were quantified by measuring the wound widths of five different wound surfaces in each group using the Image-J analysis software. The experiment was performed three times.

### Transwell migration assay

The vertical migration of mMSCs was determined using the transwell migration assay. Transwell inserts (6.5 mm diameter and 8 μm pore size; Millipore) were loaded with 1 × 10^4^ mMSCs in 200 μl of serum-free DMEM/F12, and 600 μl of DMEM/F12 supplemented with 10% FBS was added to the lower chambers. In two other groups, 50 ng/ml of CXCL12 (Abcam, Britain) was added to the lower chambers to evaluate the overexpression and suppression of CXCR7 separately. The cells were allowed to migrate at 37 °C in a humidified CO_2_ incubator for 12 h. The cells remaining on the upper surface of the filter were then removed with cotton swabs, and the cells that migrated to the lower surface were stained with crystal violet (Beyotime Institute of Biotechnology, Haimen, China) for 20 min. Stained cells from five randomly chosen fields were counted under a light microscope.

### Western blot analysis of CXCL12 protein in mMSCs

The expression of CXCL12 in mMSCs was measured using western blot analysis as previously described^18^. Briefly, total cellular protein from mMSCs was extracted in RIPA lysis buffer (Beyotime Institute of Biotechnology, Haimen, China) containing an antiprotease cocktail (1 mmol/l PMSF, 1 mmol/l NaF, and 1 mmol/l Na3VO4; US Biological Inc., Swampscott, MA, USA). Protein lysates were quantified using a BCA protein assay kit (Beyotime Institute of Biotechnology). The proteins were separated using 10% sodium dodecyl sulfate polyacrylamide gel electrophoresis (Beyotime Institute of Biotechnology) and transferred onto PVDF membranes (Millipore, Bedford, MA, USA). The membranes were blocked in Tris-1 buffer (Biosharp Biotechnology, Hefei, China) at pH 7.4 containing 0.1% Tween 20 (TBST; Sinopharm Chemical Reagent Co., Ltd., Shanghai, China) and 5% bovine serum albumin (Roche, Ltd., Basel, Switzerland) for 1 h at room temperature and were then incubated with primary antibodies to CXCL12 (1:1,000 dilution; Abcam Ltd.) or β-actin (1:3,000 dilution; Bioworld technology, Co. Ltd.) at 4 °C overnight. The blots were washed with TBST and incubated with goat anti-rabbit IgG conjugated with horseradish peroxidase (1:10,000 dilution; Zhongshan Golden Bridge Biotechnology Co. Ltd., Beijing, China) for 1 h at room temperature. Immunoreactive complexes were visualized using chemiluminescence reagents (Thermo Fisher Scientific Inc., Waltham, MA, USA).

### Measurement of surface protein and cytokines by ELISA

After 18 h of culture in a transwell assay, mMSCs and supernatants were collected and centrifuged to remove debris. Then, mMSCs were lysed by Membrane Protein Extraction Kit (Mem-PER™ Plus, Thermo Scientific, USA). CXCL12 (SDF-1α), vascular cell adhesion molecule-1 (VCAM-1), Clusters of Differentiation-44 (CD-44), matrix metalloproteinase2 (MMP2), Collagen-I, tumour necrosis factor (TNF-α) and IL-10 were measured by enzyme-linked immunosorbent assay (ELISA) kits (RayBiotech, USA; Bio-Techne, USA; Cusabio Biotech, China; ExCell Biology, China). The content of CXCL12 was determined using a semi-quantitative standard curve, and the additional CXCL12 was removed. ELISA was performed according to the manufacturer’s instructions. All samples were measured three times.

### Statistical analysis

The data were presented as the means ± standard deviation (SD). Comparisons amongst multiple groups were performed by one-way ANOVA followed by Bonferroni’s post hoc test. A *p*-value less than 0.05 was considered statistically significant.

## Results

### Lentiviral vector transduction efficiency in mMSCs

The ZsGreen-positive cell ratio was used in our study to reflect the transduction efficiency of the target gene in mMSCs. The efficiencies of the lentiviral vector transduction of MSC-OE-CXCR7, MSC-OENC-CXCR7, MSC-Sh-CXCR7 and MSC-ShNC-CXCR7 after 20 passages in mMSCs were 91.29%, 91.39%, 91.69% and 91.28%, respectively (Fig. 1a). Moreover, the RT-PCR results showed that CXCR7 mRNA expression were significantly higher in the MSC-OE-CXCR7 cells than in the MSC-OENC-CXCR7 cells (*p* < 0.05) and were significantly lower in the MSC-Sh-CXCR7 cells compared with the MSC-ShNC-CXCR7 cells (*p* < 0.05). There was no significant difference in CXCR7 mRNA expression between the MSC-Blank and MSC-OENC-CXCR7 or MSC-ShNC-CXCR7 groups (Fig. 1b). Similar results for CXCR7 protein expression were observed by flow cytometry analysis (Fig. 1c–f). These results suggest that lentivirus-mediated transduction is efficient and stable.

**Figure 1:** Long-term transgene expression efficiency in mMSCs after lentiviral vector transduction. (**a**) The mMSCs were transduced separately with pHBLV-CMVIE-CXCR7-ZsGreen-T2A-Puromycin (MSC-OE-CXCR7), pHBLV-CMVIE-ZsGreen-T2A-Puromycin (MSC-OENC-CXCR7), pHBLV-U6-ShRNA-ZsGreen-Puromycin (MSC-Sh-CXCR7) and pHBLV-U6-ZsGreen-Puromycin (MSC-ShNC-CXCR7) lentiviral vectors were cultured for 20 passages and observed with light microscopy (top) and fluorescence microscopy with green fluorescent protein (middle), 100× and 250×; the percentage of ZsGreen-positive cells were analysed by flow cytometry (bottom) at passage 20 after transduction. (**b**) Quantitative real-time PCR analysis shows CXCR7 mRNA expression in mMSCs after pHBLV-CMVIE-CXCR7-ZsGreen-T2A-Puromycin and pHBLV-U6-ShRNA-ZsGreen-Puromycin transduction. (n = 4; *p < 0.05 vs. MSC-OENC-CXCR7, ^#^ *p* < 0.05 vs. MSC-Sh-CXCR7). (**c**,**d**) FCM analysis shows CXCR7 overexpression in mMSCs after transduction. (n = 3; *p < 0.05 vs. MSC-OENC-CXCR7). (**e**,**f**) FCM analysis shows CXCR7 suppression in mMSCs after transduction. (n = 3; ^#^ *p* < 0.05 vs. MSC-ShNC-CXCR7).

### Overexpression of CXCR7 significantly improved the proliferation of mMSCs

The cell proliferation in MSC-OE-CXCR7 was significantly higher than that in the MSC-OENC-CXCR7 group (*p* < 0.001) after day 3 (Fig. 2a). In contrast, the suppression of CXCR7 (MSC-Sh-CXCR7 group) inhibited cell proliferation compared with the normal control group of suppression of CXCR7 (MSC-ShNC-CXCR7 group) (*p* < 0.05). The difference reached statistical significance on days 5 to 7 (Fig. 2b).

**Figure 2:** The effect of CXCR7 on mMSC proliferation. Cell growth curves after transduction for 7 days were evaluated by the CCK-8 assay. (**a**) The proliferation rate of the MSC-OE-CXCR7 group was significantly higher than the MSC-OENC-CXCR7 group from days 3 to 7. (n = 8; *p < 0.001 vs. MSC-OENC-CXCR7). (**b**) The proliferation rates of the MSC-Sh-CXCR7 groups were significantly lower than the MSC-ShNC-CXCR7 group from days 5 to 7. (n = 8; ^#^ *p* < 0.05 vs. MSC-ShNC-CXCR7).

### Overexpression of CXCR7 and additional CXCL12 promoted the migration of mMSCs

The effects of overexpressing CXCR7 on the horizontal and vertical migration of mMSCs were measured by the scratch and transwell assays, respectively. The scratch healing percentage increased in the MSC-OE-CXCR7 group compared with the MSC-Blank group at both 12 h and 18 h (*p* < 0.05), but it decreased in the MSC-Sh-CXCR7 group compared with the MSC-ShNC-CXCR7 group both at 12 h and 18 h (*p* < 0.05). No significant differences in the scratch healing percentage between the MSC-Blank and MSC-OENC-CXCR7 or MSC-ShNC-CXCR7 groups were observed (Fig. 3).

**Figure 3:** The effect of CXCR7 on the horizontal migration of mMSCs. The ability of mMSCs to horizontally migrate after transduction was examined using the scratch assay. The wound sites (area cleared of cells in the centre of the scratched area) were observed and photographed at 0, 12 h and 18 h, 100×. A bar graph shows the quantitative results of scratch healing. (n = 3; *p < 0.05 vs. MSC-OENC-CXCR7, ^#^ *p* < 0.05 vs. MSC-ShNC-CXCR7).

More cells migrated in the MSC-OE-CXCR7 group than in the MSC-OENC-CXCR7 group at both 12 h and 18 h (*p* < 0.05). Conversely, fewer cells migrated in the MSC-Sh-CXCR7 group at both 12 h and 18 h compared with the MSC-ShNC-CXCR7 group (*p* < 0.05). There was no significant difference in number of cells that migrated between the MSC-Blank and MSC-OENC-CXCR7 or MSC-ShNC-CXCR7 groups (Fig. 4).

**Figure 4:** The effect of CXCR7 on the vertical migration of mMSCs. Cells that migrated to the lower surface of Transwell inserts were stained with crystal violet and observed under a microscope at 12 h (**a**) and 18 h (**b**), 200×. A bar graph shows the quantitative results of cell migration. (n = 3; *p < 0.05 vs. MSC-OENC-CXCR7, ^Δ^ *p* < 0.05 vs. MSC-OE-CXCR7, ^#^ *p* < 0.05 vs. MSC-ShNC-CXCR7, ^&^ *p* < 0.05 vs. MSC-Sh-CXCR7).

Additional CXCL12 improved the vertical migration ability of mMSCs. More cells migrated in the MSC-OE-CXCR7 + CXCL12 group than in the MSC-OE-CXCR7 group at both 12 h and 18 h (*p* < 0.05), and more migration was observed in the MSC-Sh-CXCR7 + CXCL12 group than in the MSC-Sh-CXCR7 group (*p* < 0.05) (Fig. 4).

These results suggested that overexpressing CXCR7 could improve the migratory ability of mMSCs, whereas suppressing CXCR7 does the opposite.

### Overexpression of CXCR7 increased MSC-secreted CXCL12

To explore the effects of modulating CXCR7 on MSC-secreted CXCL12, we further investigated the expression of CXCL12 mRNA by qRT-PCR, the expression of CXCL12 protein in mMSCs by western blot and the concentration of CXCL12 in the supernatant of transwell chambers by ELISA. The expression level of CXCL12 mRNA was significantly higher in the MSC-OE-CXCR7 and MSC-OE-CXCR7 + CXCL12 groups than in the MSC-OENC-CXCR7 group (*p* < 0.05) but was significantly lower in the MSC-Sh-CXCR7 and MSC-Sh-CXCR7 + CXCL12 groups than in the MSC-ShNC-CXCR7 group (*p* < 0.05). Furthermore, additional CXCL12 further improved the expression of CXCL12 mRNA in MSC-OE-CXCR7 + CXCL12 and MSC-Sh-CXCR7 + CXCL12 groups compared with the MSC-OE-CXCR7 and MSC-Sh-CXCR7 groups, respectively (*p* < 0.05). However, there was no significant difference between the MSC-BLANK and MSC-OENC-CXCR7 groups (*p* > 0.05) (Fig. 5b). Similar trends were shown in CXCL12 protein expression in mMSCs by western blot analysis (Fig. 5a).

**Figure 5:** The concentration of CXCL12 in the supernatant of transwell chambers was examined using ELISA ruling out the interference of exogenous CXCL12 protein. (n = 3; *p < 0.001 vs. MSC-OENC-CXCR7, ^Δ^ *p* < 0.05 vs. MSC-OE-CXCR7, ^#^ *p* < 0.05 vs. MSC-ShNC-CXCR7, ^&^ *p* < 0.05 vs. MSC-Sh-CXCR7).

The concentration of CXCL12 in the supernatant of transwell chambers increased in the MSC-OE-CXCR7 and MSC-OE-CXCR7 + CXCL12 groups compared to the MSC-OENC-CXCR7 group (*p* < 0.05) by ELISA. Despite excluding the interference of exogenous CXCL12, the concentration of CXCL12 was still significantly higher in the MSC-OE-CXCR7 + CXCL12 group than in the MSC-OE-CXCR7 group (*p* < 0.05). CXCL12 was lower in the MSC-Sh-CXCR7 group compared with that in MSC-ShNC-CXCR7 group (*p* < 0.05). However, there was no significant difference in CXCL12 between the MSC-ShNC-CXCR7 and MSC-Sh-CXCR7 + CXCL12 groups (*p* > 0.05) (Fig. 5c).

### Overexpression CXCR7 increased MSC-expressed VCAM-1, CD-44 and MMP2

To determine the detailed mechanism by which CXCR7 regulates the proliferation and migration of mMSCs, the VCAM-1, CD-44 and MMP2 protein were measured by ELISA. VCAM-1 increased in the MSC-OE-CXCR7 and MSC-OE-CXCR7 + CXCL12 groups compared to the MSC-OENC-CXCR7 group (*p* < 0.05). The level of VCAM-1 in the MSC-Sh-CXCR7 group was lower than that in MSC-ShNC-CXCR7 group (*p* < 0.05). Additional CXCL12 further improved the VCAM-1 expression in the MSC-OE-CXCR7 + CXCL12 and MSC-Sh-CXCR7 + CXCL12 groups compared with the MSC-OE-CXCR7 and MSC-Sh-CXCR7 groups, respectively (Fig. 6a). Similar trends were shown for the concentrations of CD-44 and MMP2 (Fig. 6b,c).

**Figure 6:** The expression of VCAM-1, CD44 and MMP2 was examined using ELISA. (n = 3; *p < 0.05 vs. MSC-OENC-CXCR7, ^Δ^ *p* < 0.001 vs. MSC-OE-CXCR7, ^#^ *p* < 0.05 vs. MSC-ShNC-CXCR7, ^&^ *p* < 0.05 vs. MSC-Sh-CXCR7).

### The effect of CXCR7 on mMSC secretion of Collagen-I

To evaluate the detailed mechanism by which CXCR7 regulated the migration of mMSCs, ELISA was used to detect the Collagen-I in the supernatant of transwell chambers. However, there was no difference in Collagen-I among all groups (*p* > 0.05) (Fig. 7).

**Figure 7:** The concentration of Collagen-I in the supernatant of transwell chambers was measured using ELISA. (n = 3).

### Overexpression of CXCR7 had no significant impact on TNF-α and IL-10

To determine the effects of overexpressing CXCR7 on inflammation, the concentrations of TNF-α and IL-10 in the supernatant of transwell Chambers were measured by ELISA. There were no differences in the concentrations of TNF-α and IL-10 among all groups (*p* > 0.05) (Fig. 8a,b).

**Figure 8:** The concentration of TNF-α and IL-10 in the supernatant of transwell chambers was measured using ELISA. (n = 3).

## Discussion

Great interest has been shown in MSC therapy for a wide variety of clinical domains, such as moderate-to-severe ARDS^19–22^. However, its therapeutic efficiency depends on the proliferation and migration of MSCs to a target tissue^23^. The major findings of the present study were as follows: (1) the overexpression of CXCR7 significantly improved the proliferation and migration of mMSCs; (2) the positive feedback regulation of CXCL12 and the increased expression of VCAM-1, CD44, and MMP2 could be attributed primarily to the improved homing of mMSCs when overexpressing CXCR7; and (3) Overexpression of CXCR7 does not seem to exert major impact on inflammation.

The third generation of self-inactivation (SIN) human immunodeficiency virus type 1 (HIV-1) was chosen as a vector of target gene overexpression in this study. Several studies have confirmed that HIV-1-based SIN lentivirus vectors sustain high levels of transgene expression in human embryonic stem cells, although their application in MSCs is still unknown^24,25^. Therefore, lentivirus vectors pHBLV-CMVIE- ZsGreen-T2A-Puromycin and pHBLV-U6-ZsGreen-Puromycin were successfully constructed for gene transfection and interference, which contains CMV promoter and U6 promoter.

Improving the proliferation and migration of MSCs to a target tissue is the key issue for improving the efficiency of the therapy. A concentration gradient of CXCL12 can specifically regulate different effects of chemotaxis in stem cells^26–28^. In a previous study, CXCR4 was considered the unique receptor of CXCL12 and was shown to play an important role in chemotaxis^11,29^. Balabanian and Burns found that there was another binding site of CXCL12, named RCD1 (CXCR7) in 2006. The affinity of CXCR7 to CXCL12 is 10 times greater than that of CXCR4^11^. However, the lower cell surface expression of CXCR7 than of CXCR4 has seriously restricted the role of the CXCL12/CXCR7 axis on the migration of mMSCs. The present study demonstrates that the overexpression of CXCR7 significantly improved and that the low expression of CXCR7 decreased the proliferation and migratory ability of mMSCs. Additional CXCL12 was added to simulate inflammation microenvironments, which further increased the migratory ability of mMSCs. Our results suggest that the overexpression of CXCR7 have a positive effect on MSC proliferation and migration. However, Liu *et al*.^30^ found that CXCR7 was shown to have no influence on MSC migration in renal ischaemia/reperfusion injury models. Gheisari *et al*.^31^ found that CXCR7-transfected MSCs were trapped in the lungs, whereas native MSCs home very rarely to kidneys and bone marrow. In addition, the activation of CXCR7 may improve the migration of colorectal cancer cells in the lung but not in the liver^9^. Thus, it is suspected that MSCs overexpressing CXCR7 may have organ specificity, especially in the lungs.

Paracrine adhesion factors have been proposed to be the primary mechanism for MSC migration^32^. To explore the detailed mechanism of increased migration of mMSCs by overexpressing CXCR7, the levels of VCAM-1, CD44, MMP2 and Collagen-I, which are important MSC paracrine factors that regulate the vascular adhesion of MSCs^33,34^, were measured in the supernatant of transwell chambers. However, VCAM-1, CD44, and MMP2 increased and decreased significantly after overexpression and suppression of CXCR7, respectively. It has been demonstrated that blocking VCAM-1 by its antibody significantly reduced the migration of MSCs^28^. Further, CD44 and MMP2 play important roles in the migration of MSCs. Thus, this study showed that the increased mMSC secretion of VCAM-1, CD44, and MMP2 is one of the primary mechanisms related to mMSC migration that are promoted by the overexpression of CXCR7.

In previous studies, the expression of CXCL12 increased significantly in injured and hypoxic tissues^10,35,36^. Thus, additional CXCL12 was added to the lower chambers of transwell assays to simulate the microenvironment of injured and hypoxic tissues. We found that the overexpression of CXCR7 in mMSCs not only improved their migration and proliferation but also increased their CXCL12 secretion. The mechanism is possibly described based on the following two phenomena. On one hand, more CXCL12 combined with its ligand CXCR7 when CXCR7 was overexpressed in mMSCs, which may have increased the ability of these cells to migrate. The supplemented CXCL12 may combine with more CXCR7 and CXCR4 on mMSCs in a positive feedback loop, which was also reported in Wang’s study^37^. On the other hand, the high expression of CXCR7 may activate the CXCL12/CXCR7 axis, thus making mMSCs secrete more CXCL12. It was supported by the increasing protein and mRNA level of CXCL12. If true, this would be a novel discovery, however, further study is needed.

One concern is that gene transfection may influence the function of mMSCs or promote inflammation^38,39^. There were no significant changes in TNF-α or IL-10 among the groups in the supernatant of transwell chambers in this study^40^. Our results may prove that MSCs that migrate after CXCR7 gene transduction are not associated with inflammation, which ensures the safety of overexpressing CXCR7 in mMSCs that are transferred to animals for further research.

One limitation of our study should be noted. In our experiments, lipopolysaccharide was not added, which cannot simulate endotoxin-related injury. This will be explored further in follow-up studies.

In conclusion, we demonstrated that lentiviral vector transduction successfully facilitated the sustained and efficient gene modification of CXCR7 in mMSCs. The overexpression of CXCR7 significantly improved the proliferation and migration of mMSCs without inducing inflammation. The mechanism is the positive feedback regulation of CXCL12 and is related to the increased expression of VCAM-1, CD44, and MMP2 but not Collagen-I. Our results provide a potential method for improving the treatment effectiveness of mMSCs by overexpressing CXCR7. Further animal research will be necessary to explore the treatment effects of overexpressing CXCR7 in mMSCs.
